This article has been retracted.

# Male breast cancer: thirteen years experience of a single center

**DOI:** 10.1186/1477-7800-6-4

**Published:** 2009-02-05

**Authors:** Sami Akbulut, Ilker Arer, Alper Kocbiyik, Mahmut Can Yağmurdur, Hamdi Karakayalı, Mehmet Haberal

**Affiliations:** 1 Department of Surgery, University Hospital of Baskent, Ankara 06490, Turkey; 2 Department of Pathology, University Hospital of Baskent, Ankara 06490, Turkey

## Abstract

**Background:**

This retrospective study analysed the epidemiological, clinical, and therapeutic profiles of breast cancer in males.

**Methods:**

We report our experience at the Hospital of the University of Baskent, where 20 cases of male breast cancer were observed and treated between 1995–2008.

**Results:**

Median age at presentation was 66,7 ± 10,9 years. Average follow-up was 63 ± 18,5 months. The main presenting symptom was a mass in 65% of cases (13 patients). Ýnvasive ductal carcinoma was the most frequent pathologic type (70% of cases).

**Conclusion:**

Male breast cancer patients have an incidence of prostate cancer higher than would be predicted in the general population. Cause of men have a higher rate of ER positivity the responses with hormonal agents are good.

## Background

Male breast cancer(MBC) is infrequent; it accounts for 0,8% of all breast cancers, less than 1% of all newly diagnosed male cancers, and 0,2% of male cancer deaths. The median age at diagnosis is 68 years, 5 years older than in women. [1-4].

The aim of this retrospective study was to present our results and analyse the epidemiological, clinical, and therapeutic profiles of this disease in 20 cases treated in our unit between1995 and 2008.

## Patients and methods

Twenty male patients with breast cancer were treated at our University between 1995 – 2008. median age at presentation was 66,7 ± 10,9 years (range 56–90 years).

## Results

Ýn two cases the disease was diagnosed incidentally after CT scan of the thorax for other conditions. In three cases, prostate cancer was conicident, renal cell cancer was present in one case. The disease developed after renal transplantation in one case, Kaposi sarcoma in one case. There was a family history of breast cancer in two cases.

Fourteen patients (70%) had a left-sided breast cancer and six patients (30%) had a right-sided tumour. The median follow-up was 63 ± 18,5 months (range: 4–149 months).

Three patients developed local recurrence (Chest wall in one patient, axillary lymph nodes in two patients).

The presenting clinical symptom was a mass in 13 of cases. Pain was the second complaint in 4 of cases. The tumour associated with breast ulceration in 2 of cases and a bloody nipple discharge in one of cases (graphic 1). Upper outer quadrant masses were present in 80% of cases, a retroareolar mass in 10%, and inner quadrants mass in 10%.

Bone pain was observed in one patient, related to presence of metastases. The diagnosis was confirmed by excisional biopsy in 75% cases and tru-cut biopsy in 25% cases.

The type of surgical procedure and tumors size was showed in Figure 1 and 2.

**Figure 1:** **Distribution of patients according to the operation type**. MRM: Modified radical mastectomy, Q+AND: Quadranectomy + axillary node dissection, L+AND: Lumpectomy + axillary node dissection, RM: Radical mastectomy.

**Figure 2:** **Dsitribution of patients according to the tumour size (T)**. Tis: carcinoma insitu.

Pathogical analysis of the specimens revaled infiltrating ductal carcinoma (IDC) in 70% (14 cases), which one of has mucinous carcinoma togetherness, ductal carcinoma in situ (DCIS) in 25% (5 cases), and one case of coexistent apocrine carcinom and micropapillary carcinoma [5]. One of the IDC was associated with primary unkown adenocarcinoma. Pathological characteristics were showed in Figure 3

**Figure 3:** **Invasive apocrine carcinoma with desmoplastic stroma (H&E, ×100)**. (**A1**), Estrogen receptor shows strong positivity (approximately %80 of the tumor cells) (**A2**), Progesteron receptor reveals the same features with ER (**A3**), Cytoplasm expression of HER2/neu, no membranous stainning (**A4**), Diffuse stainning for gross cystic disease fluid protein (GCDFP15) (**A5**), Invasive ductal component of the invasive mucinous carcinoma at the perifery of the tumor (H & E, ×40) (**B1**), H & E sections (×100) (**B2**), Approximately the whole of the tumor cells shows estrogen receptor positivity (B3), The same stainning features for progesteron (B4), There is no HER2/neu expression, whereas positive control reveals membranous staining (left corner) (B5), Tumor cells arranged in morula-like clusters, reffered to as an ''exfoliative appearance'' (H & E, ×100) (**C1**), There is no estrogen receptor positivity, whereas positive control reveals staining (left corner) (**C2**), Approximately 50% of the tumor cells show progesteron receptor positivity (moderate staining) (**C3**), There is no HER2/neu expression, whereas positive control reveals membranous staining (left corner) (**C4**), There is stainning for EMA (epithelial membran antigen) at the perifery (**C5**).

### Lymph node ınvolvement

Axillary lymph nodes contained metastasis in 6 of the cases. Five of 6 cases had more than four lymph nodes involved. One of 6 cases had nipple areola complex invasion. Four of cases had positive lymph nodes with extra-capsular extension.

### Hormone receptors

Fourteen cases had 30% to 100% positive ostrogene, progestrogene receptors. Three case had only positive ostregene receptor. In three patients examination of hormone receptore was not done

Because the operations of these 3 patients was done between 1995–1998 and at that years receptor scanning was not been performed routinely.

Examination of c-erb-2 oncoprotein was done in 15 patients. There was not any staining with c-erb b2 except one case who has apocrin carcinoma.

### Treatment

Adjuvant radiation therapy with an average dose of 50 Gy was given to all of the patients who had axillary lymph node metastasis and to whom performed breast sparing surgery. In addition, tamoxifen therapy was also given if the hormone receptors were positive.

Only hormonal therapy was given in one case who had an apocrine carcinoma, and had 80% positive hormone receptor and categorized as T_2_N_0_M_0_.

Adjuvant radiation therapy, chemotherapy and hormonal therapy was given in patient(T_2_N_0_M_0_) who had IDC and mucinous carcinoma together and in patient who had a chest wall invasion.

### Outcome

After the first therapy protocole the patients were taken to a 6 month follow-up. Only 2 cases, the cases with bone and lung metastasis, were lost. Of the cases with extracapsullary invasion two of them and n the patient with T4 tumour (in the chest wall) showed local recurrence. Radio- and chemotherapy were given to these cases with a difference of excision addition to the chest wall recurrence. At the end of the six month, local recurrences regressed totally. All of the alive 18 cases came to the control in the last year. The doses of agents placed in the therapy protocole of immunosuppressive patients, were reduced to minimum. None of them shows pathological evidence belong to metastasis or local invasion.

## Discussion

MBC is an uncommon disease, which presents mostly in the latter decades of life. It represents less than 1% of all malignancies in men and is responsible for 0,1% of male cancer deaths [2]. It behaves similiar to female breast cancer in most cases [6]. In our clinic incidence ratio is 2, 9:100 which is more than literature [7].

Men have a higher rate of ER positivity, which accounts for good responses with hormonal agents as in our study. We used only tamoxifen in all ER positive, DCIS cases. We used tamoxifen combined with radiotherapy in ER positive, IDC cases. The prevalence of MBC increases with age, with a mean age of 60–65 years at presentation [8]. Risk factors include increasing age, radiation exposure, and factors related to abnormalities in estrogen and androgen balance, including testicular disease, infertility, obesity, and cirrhosis. Risk factors related to a genetic predisposition include Klinefelter's syndrome, family history, and *BRCA *gene mutations, particularly *BRCA2 *mutations. Gynecomastia is not a risk factor [9].

Male breast cancer patients have an incidence of prostate cancer higher than would be predicted in the general population; this risk factor has implications for prostate cancer screening. In a recent study of Lee UJ et all, 12 of 69(17%) patients with male breast cancer also had a diagnosis of prostate cancer [10]. In our study 3 of 20(15%) patients had breast cancer with prostate cancer.

Breast cancer occurred in two patients with immunosuppressive disorders in our series.

MBC is usually diagnosed at an advanced stage, with a typical subareolar mass associated with axillary lymph nodes and pain [11,12].

The male breast contains only ductal tissue, hence, most MBCs are of the ductal type. Histologically, 90% of male breast cancers are invasive ductal carcinomas. Approximately 80% are ER positive, 75% are PR positive, and 35% overexpress HER-2/neu. The remaining 10% are DCIS. Given the absence of terminal lobules in the normal male breast, lobular carcinoma, both invasive and in situ, is rarely seen [3,4].

The most common surgical treatment is modified radical mastectomy with axillary node dissection. Adjuvant radiotherapy has an important role in reducing the risk of local recurrence in large tumors, lymph node and muscle involvement [13]. Tamoxifen is the most widely used adjuvant therapy, because it improves survival. It may be associated with more limited side effects in men than in women, like decreased libido, weight gain, hot flushes, mood alterations, depression, insomnia and deep vein thrombosis. There is no evidence that chemotherapy improves long term survival. Chemoterapy may be useful in node positive and locally advanced disease. The use of adjuvant RT has not been conclusively proven to reduce local recurrence.

Prognostic factors in male breast cancer are the same as in female breast cancer and include nodal involvement, tumor size, histologic grade, and hormone receptor status. When matched for age and stage, survival is similar to that in women. Poor prognosis is attributed to old age, axillary lymph node metastases(>4) and negative hormone receptors [13,14].

## Competing interests

We confirm, none of the authors listed in this manuscript have any financial or other conflicts of interest to disclose.

## Authors' contributions

SA, MCY and HK contributed writing the article and review of the literature as well as undertaking a comprehensive literature search; SA and IA contributed design and manuscript preparation; AK provided the histopathologycal information.
